This article has been retracted.

# Tumor-associated fibroblasts derived exosomes induce the proliferation and cisplatin resistance in esophageal squamous cell carcinoma cells through RIG-I/IFN-β signaling

**DOI:** 10.1080/21655979.2022.2076008

**Published:** 2022-05-19

**Authors:** Yayun Cui, Shu Zhang, Xiaohan Hu, Fei Gao

**Affiliations:** a Department of Cancer Radiotherapy, The First Affiliated Hospital of USTC, Division of Life Sciences and Medicine, University of Science and Technology of China (Anhui Provincial Cancer Hospital), Hefei, Anhui, China; b Department of Gastroenterology, Shandong Cancer Hospital and Institute, Shandong First Medical University and Shandong Academy of Medical Sciences, Jinan, Shandong, China; c Laboratory of Medicine, Nanjing Drum Tower Hospital, Nanjing University Medical School, Nanjing, Jiangsu, China; d Department of Radiology, The First Affiliated Hospital of USTC, Division of Life Sciences and Medicine, University of Science and Technology of China (Anhui Provincial Cancer Hospital), Hefei, Anhui, China

**Keywords:** ESCC cells, TAFs, exosomes, cisplatin, chemosensitivity

## Abstract

Esophageal squamous cell carcinoma (ESCC) is a common type of malignant cancer. There is growing evidence suggesting that exosomes may participate in the cellular communication of tumor-associated fibroblasts (TAFs). However, the cisplatin resistance of TAF-derived exosomes to ESCC cells remains to be further studied. Exosomes were isolated from TAFs and characterized with Western blot and TEM assays. ESCC cell lines (TE-1 and KYSE-150) were incubated with TAFs-derived exosomes. To explore the biological function of TAF-derived exosomes in ESCC cell proliferation, apoptosis, and chemosensitivity, we conducted MTT assays and Flow Cytometry. The effects *in vivo* were also verified via Xenograft mice models. We found that TAFs-derived exosomes led to enhanced cell proliferation and reduced apoptosis of cells, accompanied by increased expression of RIG-I/IFN-β, and TAFs derived exosomes may affect the chemosensitivity to cisplatin via RIG-I/IFN-β signaling in ESCC. Taken together, ESCC cells could communicate with TAFs cells via TAFs-derived exosomes. Our findings might represent a novel mechanism involved in ESCC and may provide a potential biomarker for ESCC.

## Highlights

- TAFs derived exosomes induced proliferation and inhibited apoptosis of ESCC cells.
- TAFs derived exosomes induced the activation of RIG-I/IFN-β signaling in ESCC cells.
- TAFs derived exosomes affected the chemosensitivity of TE-1 cells to cisplatin.
- ESCC cells communicated with TAFs cells via exosomes.

## Introduction

Esophageal squamous cell carcinoma (ESCC) is a common malignant cancer type worldwide [1,2]. Due to the early transferability of ESCC, the 5-year overall survival rate for ESCC patients remains below 20% [2]. With the rapid increase in ESCC incidence and mortality, it is estimated that more than 1 million new cases will suffer from ESCC in the next decade [3]. Current clinical treatment methods for ESCC patients include surgery and adjuvant chemotherapy. Cisplatin is the basic drug used in the treatment of ESCC. However, cisplatin resistance has become more and more common and drug resistance remains a major obstacle to cisplatin therapy in patients, which usually leads to relapse or even death [4]. Therefore, further researches are required to elucidate the pathological mechanisms of ESCC development and drug resistance, which may help to formulate effective therapeutic strategies for ESCC.

Tumor microenvironment (TME) is formed by cancer cells and extracellular matrix, including tumor-associated fibroblasts (TAFs), macrophages, etc., which affects the process of tumor growth, drug resistance, and metastasis [5–9]. TAFs are a crucial part of the TME and they are vital to the generation of tumor chemotherapeutic drug resistance. For example, Shintani et al. found that IL-6 from TAFs induces chemoresistance by enhancing epithelial mesenchymal transition in non-small cell lung cancer cells [10]. Smooth muscle actin (α-SMA) is one of the markers that identify the TAFs. α-SMA presents a higher expression level in TAFs [11–13]. Evidence has shown that cross-talk between tumors and TAFs can mediate tumor growth, metastasis, invasion, and other key oncology behaviors [14,15]. However, how TAFs induce drug resistance remains to be further investigated.

Exosomes are membrane vesicles approximately 30–100 nm in diameter that can be secreted by nearly all cells into the extracellular environment [16,17]. They are generally characterized by cell surface tetraspanin proteins: CD9, CD63, and CD81 [18]. Exosomes can deliver diverse types of molecules to target cells, including proteins, lipids, and nucleic acids, through which they can mediate intercellular communications [19,20]. Growing evidence indicates that exosomes can work as critical intercellular messengers to promote tumor development [17,21,22]. A recent study illustrates that ESCC-released exosomes can induce phenotypic changes in T cells and monocytes/fibroblasts, which may consequently contribute to tumor progression [14]. However, it has not been fully understood how ESCC cells communicate with fibroblasts via exosomes.

Combined with the above studies, we hypothesized that ESCC cells could induce cisplatin resistance through crosstalk with TAF via exosomes. Therefore, the aim of this study was to investigate the effects and mechanism of TAFs-released exosomes on the proliferation and cisplatin resistance of ESCC cells *In vitro* and *In vivo*. We found that TAFs-derived exosomes induced the cell proliferation and inhibited the cell chemosensitivity to cisplatin in ESCC via the RIG-I/IFN-β signaling pathway. These findings help us to better understand ESCC mechanisms and might provide a new therapeutic idea for ESCC patients.

## Material and methods

### Cell culture

TE-1 and KYSE-150 cells were obtained from the Shanghai Cell Bank of Chinese Academy of Sciences. Cells were cultured in RPMI-1640 medium (Invitrogen, Carlsbad, USA) at 37°C in a 5% CO_2_ incubator. Medium was supplemented with 10% FBS (Invitrogen, Carlsbad, USA) and 1% (w/v) penicillin/streptomycin (Sigma-Aldrich, MO, USA).

### *Isolation and characterization of TAFs* [23]

TAFs were isolated from ESCC tumor tissues. This study was approved by the ethics committee of Anhui Provincial Cancer Hospital (2019-FLK-04). Before collecting tumor samples, written informed consent was obtained from each patient (Clinical data for each individual human subject were shown in supplementary file clinical information). Tissues were cut into small pieces of 1–3 mm under aseptic conditions. Next, digested with 1 mg/mL collagenase I (Sigma) were used to digest tissue fragments in a cell culture incubator. Took it out every 0.5 h and shook it gently until the tissue mass was completely digested and dispersed. Then, after filtering through a 200-mesh filter and centrifuging, the cell pellets were inoculated into the culture flask. After the cells have been cultured for 30 min, replace with the fresh medium to remove non-adherent cells. Finally, TAFs isolated from ESCC tissues were cultured in RPMI 1640 medium. The specific marker α-SMA was detected by the flow cytometry to confirm the characteristics of fibroblasts and exclude epithelial cell contamination [24]. The TAFs used in the experiment were all less than 8 generations. TAFs-released exosomes were incubated with ESCC to study the function of exosomes.

### Exosome isolation and characterization

Exosomes were obtained using differential centrifugation as described previously [25]. Condition media from TAFs cells were collected and centrifuged at 300, 1200, and 10,000 g for 10, 20, and 30 min, respectively. Then cells, cell debris, and large particles were removed, respectively. ExoPrep reagent was then added to the supernatant on ice for 1 h. Then the mixture was centrifuged at 10,000 and 1500 g for 20 and 2 min, respectively. Subsequently, 100 µl PBS was used to re-suspended the exosome pellet. The exosome samples were assessed using Western blot and transmission electron microscope as described below.

### Transmission Electron Microscopy (TEM)

TEM was conducted to identify the purified exosome [26]. Carbon-coated copper grids (200 mesh) were performed to adsorb exosomes (10 µl) for 1 min in a dry environment. Then distilled water was employed to wash the grids for 2 min. This was followed by negative staining with 2% uranyl acetate solution for 1 min. Finally, the air-dried grids were observed by TEM at 80 kV.

### *Cell proliferation assay* [27]

TE-1 cells (5 × 10^4^) were planted in 96-well plates per well. Then exosomes were added for different times (12, 24, 48 h). Next, 20 µl MTT solution (Sigma) was added to each well. Subsequently, the cells were continued incubating for 4 h. After that, 100 µl DMSO (Sigma) was applied to dissolve intracellular purple formazan crystals. Finally, the OD value was measured at 490 nm to evaluated cell proliferation.

### Real-time quantitative PCR (RT-qPCR)

TRIZOL reagent was performed to obtain total RNA (Thermo Fisher Scientific). It is subsequently transcribed into cDNA via PrimeScript™ RT reagent Kit (TaKaRa). SYBR® Premix Ex Taq™ kit (TaKaRa) was applied to conduct RT-qPCR reactions on ABI 730 RT-qPCR System (Applied Biosystems). The thermocycling profiles were as follows: 95°C for 30 s, then 40 cycles of 95°C for 5 s and 60°C for 30 s. The 2^−ΔΔCt^ method was performed to calculate the mRNA expression that was normalized to the Glyceraldehyde 3-phosphate dehydrogenase (GAPDH) [28]. Primers are listed in Table 1.

**Table 1.** The primer sequences of RIG-1, IFN-β and GAPDH for RT-qPCR

Gene	Primer sequence (5′–3′)
RIG-1	F: GACCCTCCCGGCACAGA R: TCAGCAACTGAGGTGGCAATC
IFN-β	F: AACAAGTGTCTCCTCCAAATTGC R: GCAGTATTCAA GCCTCCCATTC
GAPDH	F: CGAGCCACATCGCTCAGACA R: GTGGTGAAGACGCCAGTGGA

### *Western blot* [29]

Ice-cold RIPA lysis buffer was applied to isolate protein from cells (Beyotime). Then, A Pierce® BCA Protein Assay Kit (Thermo Fisher Scientific) was employed to assess the protein concentration. Next, 10% SDS-PAGE was used to separated protein after denaturation by boiling water bath. Subsequently, the proteins were transferred onto PVDF membranes and then blocked with 5% nonfat milk in tris-buffered saline (TBS). Primary antibodies were added and incubated at 4°C overnight. The next day, the washed membranes were incubated with secondary antibodies conjugated with HRP at room temperature for 60 min. Finally, a ECL Reagent Kit (Thermo Fisher Scientific) and ChemiDoc™ XRS+ imaging system (Bio-Rad) were applied to visualize the protein bands.

### Flow cytometry

Annexin V-PI Apoptosis Detection kit (BD Biosciences) was performed to assess cell apoptosis [24]. In brief, cells were washed and re-suspended in a cold binding buffer. Then, cells were stained with Annexin V/FITC and PI for 15 min in darkness, and subjected to flow cytometry analysis (BD Biosciences). Finally, the apoptosis rate was analyzed by CellQuest software (BD Biosciences).

### Xenograft tumor models

Fifteen BALB/c-nu/nu male nude mice at 4–6 weeks were obtained from Animal Center (Nanjing Medical University, Nanjing, China). There are five mice in each group. For xenograft tumor models [26], 2 × 10^6^ TE-1 cells were suspended in PBS and then subcutaneously injected into the right flank of the mice. Seven days after cell injection, normal saline, cisplatin (5 mg/kg/5 days) or exosome (100 μg/mice/3 days) were intraperitoneally injected into mice. Mice were sacrificed in a CO_2_ chamber (flow rate<30% volume per min) for 7 minutes after anesthesia with isoflurane on day 28. Tumor tissue was excised and weighed when the animal was finally confirmed to be dead. All experimental studies were performed according to animal protocols approved by the National Institutes of Health Guide for the care and use of laboratory animals and the ethical committee on animal research of Anhui Provincial Cancer Hospital (Anhui, China) (2019-FLK-04).

### Statistical analysis

GraphPad Prism software was applied to analyze the results. Data were present as means ± standard deviation. Student’s t-test was performed to analyze the statistical significance. *p* < 0.05 is considered statistically significant.

## Results

This study aimed to explore the effects and mechanism of TAFs-exosomes on ESCC cell proliferation and drug resistance. We found that co-culture of ESCC cells with exosomes isolated from TAFs resulted in enhanced cell proliferation and decreased apoptosis, as well as increased cell resistance to cisplatin. Mechanistic studies revealed that exosomes increased the expression of RIG-I/IFN-β in cells. However, knockdown of RIG-I inhibited cell proliferation and promoted apoptosis. In addition, *In vivo* experiments also demonstrated that exosomes inhibited the sensitivity of ESCC cells to cisplatin. In conclusion, TAFs-exosomes transported RIG-I to activate the RIG-I/IFN-β signaling pathway, thereby promoting cell proliferation and cisplatin resistance. Targeting RIG-I/IFN-β axis may provide promising biomarkers and new strategies for the clinical treatment of ESCC chemoresistance.

### Isolation and identification of TAFs exosomes

Firstly, TAFs were isolated from ESCC tissues. Flow cytometry was applied to identify the biomarkers of separated cells, including α-SMA, CD34, and CD45. The cells mainly showed the characteristics of α-SMA (+), CD34 (-), and CD45 (-). The positive rate of α-SMA is greater than 99%, suggesting that it had the characteristics of fibroblasts. On the other hand, CD34 and CD45 were almost not expressed, confirming that they were not derived from endothelial and myeloid cells (Figure 1(a)). Exosomes derived from TAFs were isolated by sequential centrifugation and ExoPrep reagent. The isolated exosomes were characterized by TEM and Western blot analysis. In TEM analysis, we observed intact circular particles, ranging in diameter from about 30 to 150 nm (Figure 1(b)). In addition, we also found that the expression of exosome-specific markers CD9, CD63, and CD81 in the vesicles was highly positive (Figure 1(c)).

**Figure 1.** Isolation of exosomes from TAFs cells.(a) Flow cytometry was used to detect the expression of α-SMA, CD34, and CD45. (b) Representative TEM images of exosomes derived from TAFs cells showing morphology and size range. Scale bar = 200 nm. (c) Representative Western blot showing the expression of exosome markers (CD63, CD9, and CD81).

### TAFs derived exosomes induce proliferation and inhibit apoptosis of ESCC cells

We hereby examined the function of exosomes after incubation with TE-1 and KYSE-150 cells. MTT assay revealed that exosomes promoted cell proliferation. And after 48 h of culture, we observed that cell proliferation was obviously increased (Figure 2(a)). Flow cytometry revealed that exposure to exosomes led to the decrease of apoptosis (Figure 2(b)). Moreover, results of Western blot analysis showed that exosomes promoted the anti-apoptosis protein (Bcl-2) and inhibited the pro-apoptosis protein (Bax and cleaved-Caspase-3) (Figure 2(c)). The above results all showed that exosome regulated the proliferation and apoptosis of ESCC cells.

**Figure 2.** Exosomes induce proliferation and inhibit apoptosis of ESCC cells.(a) MTT assay to examine the cell proliferation. The data were shown as the optical density measured at 490 nm. (b) Flow cytometry was applied to assess cell apoptosis. (c) Western blot of Bcl-2, Bax and caspase-3. *, *p* < 0.05; **, *p* < 0.01.

### TAFs derived exosomes induce the activation of RIG-I/IFN-β signaling in ESCC cells

Next, the molecular mechanism by which TAFs-derived exosomes induced ESCC cell proliferation and inhibited apoptosis RIG-I were evaluated. We found that exosomes had significantly enhanced the expressions of RIG-I and IFN-β on both mRNA (Figure 3(a)) and protein (Figure 3(b)) levels in ESCC cells. These indicated that TAFs-exosomes may participate in the regulation of proliferation and apoptosis of ESCC cells by activating RIG-I/IFN-β signaling.

**Figure 3.** TAFs derived exosomes affect the chemosensitivity of ESCC cells to cisplatin via RIG-I/IFN-β signaling.(a) RT-PCR analysis of RIG-I/IFN-β. (b) Western blot analysis of RIG-I/IFN-β. **, *p* < 0.01; ***, *p* < 0.001.

### TAFs derived exosomes reduce the chemosensitivity of ESCC cells to cisplatin

Furthermore, the function of TAFs-derived exosomes on the chemosensitivity of ESCC cells to cisplatin was evaluated. We found that cisplatin treatment significantly suppressed the proliferation while enhancing the apoptosis in TE-1 and KYSE-150 cells (Figure 4(a,b)). However, TAFs exosomes partially abolished these effects (Figure 4). These results revealed that TAFs-exosomes decreased the chemosensitivity of ESCC cells to cisplatin.

**Figure 4.** TAFs derived exosomes affect the chemosensitivity of ESCC cells to cisplatin.(a) MTT assay was employed to examine the cell proliferation. (b) Flow cytometry was applied to analyze cell apoptosis. *, *p* < 0.05; **, *p* < 0.01.

### TAFs derived exosomes inhibit the chemosensitivity of ESCC cells to cisplatin via RIG-I/IFN-β signaling

Likewise, we further investigated whether TAFs-exosomes affected cisplatin resistance of ESCC cells via RIG-I/IFN-β signaling. The results showed that while cisplatin markedly decreased the expressions of RIG-I and IFN-β both on mRNA (Figure 5(a)) and protein (Figure 5(b)) levels, whereas TAFs-derived exosomes partially restored the down-regulation of RIG-I and IFN-β caused by cisplatin. Next, we performed rescue experiments by knockdown the expression of RIG-I in TAFs-exosomes. RT-qPCR (Figure S1(a)) and western blot (Figure S1(b)) results showed that knockdown of RIG-I in TAFs-exosomes inhibited the up-regulation of RIG-I and IFN-β mRNA and protein expressions in cells caused by exosomes (Figure S1). Finally, we also examined the effect of RIG-I knockdown on ESCC cell proliferation, apoptosis, and cisplatin resistance. As mentioned earlier, cisplatin suppressed cell proliferation (Figure S2(a)) and enhanced apoptosis (Figure S2(b)), while TAFs-exosomes partially resisted this cisplatin effect. Surprisingly, knockdown of RIG-I reversed this cancer-promoting effects of TAFs-exosomes again, making cell proliferation re-lessened (Figure S2(a)) and apoptosis re-heightened (Figure S2(b)). Taken together, these results confirmed that TAFs derived exosomes regulated ESCC cell proliferation, apoptosis, and cisplatin resistance through the RIG-I/IFN-β pathway.

**Figure 5.** TAFs derived exosomes affect the chemosensitivity of ESCC cells to cisplatin via RIG-I/IFN-β signaling.(a) RT-PCR analysis of RIG-I/IFN-β. (b) Flow cytometry was applied to assess cell apoptosis. *, *p* < 0.05; **, *p* < 0.01.

### TAFs derived exosomes suppress the cisplatin chemosensitivity *in vivo*

Finally, we performed *in vivo* experiments to assess the effects of TAFs-derived exosomes on the chemosensitivity of ESCC cells to cisplatin. It can be indicated that TAFs-derived exosomes markedly increased the size and weight of the tumor in mice inhibited by cisplatin treatment (Figure 6(a)). Moreover, TAFs derived exosomes also increased expressions of RIG-I and IFN-β in xenograft tumor tissues (Figure 6(b)).

**Figure 6.** TAFs derived exosomes affect the cisplatin chemosensitivity *in vivo.*(a) Images and tumor weight of the xenograft tumors. (b) Western blot analysis of RIG-I/IFN-β. *, *p* < 0.05; **, *p* < 0.01.

## Discussion

TAFs are important parts of the tumor microenvironment. Exosomes are also important mediators in crosstalk between TAFs and tumors. Recent studies implied that TAF-derived exosomes are vital to the development and chemoresistance of cancer cells [30]. For example, a study reported that TAFs-derived exosomes can activate the TGFβ1 signaling to promote epithelial-mesenchymal transition of ovarian cancer cells [31]. Another study showed that miR-21 derived from TAF-exosomes has been proved to accelerate oxaliplatin resistance in colorectal cancer [32]. Moreover, TAFs-exosomes promote RNA stability and XIAP transcription by transporting the lncRNA SNHG12 to bind to HuR, thereby enhancing DDP resistance in lung cancer [33]. Zhou *et al*. found that TAF-derived exosomes transported circZFR to hepatoma cells, thereby promoting their development and cisplatin chemoresistance [34]. However, the function of TAF-derived exosomes in ESCC cisplatin resistance has not been elucidated. Therefore, we investigated whether TAFs-derived exosomes can influence ESCC cells and explored the possible mechanisms.

We isolated and identified TAFs-derived exosomes in this research. The results showed that the α-SMA positive rate of fibroblasts isolated from ESCC tissues was greater than 99%, along with CD34 and CD45 almost not expressed, which suggested that the cells have fibroblast characteristics. Meanwhile, the exosomes isolated from TAFs range in diameter from 30 to 150 nm, and highly express exosome specific marker proteins (CD63, CD9, CD81). Our data confirmed that we have successfully isolated exosomes from TAFs.

Exosomes can mediate cellular information communication and subsequently regulate cell biological functions. For example, exosome-derived miR-154-5p attenuates ESCC progression and angiogenesis by targeting KIF14 [35]. However, the mechanism of how exosomes crosstalk with TAF to mediate ESCC cell proliferation and drug resistance has not been fully elucidated and needs to be further explored. Thus, we addressed the questions of whether TAFs-derived exosomes have effects on ESCC cells. TAF-derived exosomes obviously induced proliferation and reduced apoptosis in TE-1 and KYSE-150 cells. Moreover, Bcl-2, Bax, and caspase-3 are identified as apoptosis-related proteins [36]. After incubation with exosomes, Bcl-2 expression was significantly increased while Bax and caspase-3 expression was significantly decreased in TE-1 and KYSE-150 cells. Taken together, the results suggested that TAFs-derived exosomes can affect the cell proliferation and apoptosis of TE-1 and KYSE-150 cells *in vitro*.

Furthermore, evidence has shown that the signaling RIG-I/IFN-β is involved in cell proliferation and apoptosis [37,38]. Recently, various studies suggested that RIG has a dual role in cancer. For example, the average expression of RIG-I was highly increased in pancreatic ductal adenocarcinoma tissues, which could promote the cells’ growth and link to a lower survival rate [39]. In contrast, RIG-I is clearly decreased in liver cancer. prognosis [40]. Quercetin inhibited cell development of melanoma tumor cells B16 *in vitro* through RIG-I/IFN-β signaling [41]. These studies indicate that RIG-I is related to tumor development and resistance to radiotherapy and chemotherapy. In our study, RIG-I/IFN-β signaling in ESCC cells was activated by TAFs-derived exosomes, which explained that the pro-proliferative effect of TAFs-derived exosomes may be partially dependent on the RIG-I/IFN-β signaling pathway.

Exosomes were known to regulate the chemosensitivity of different types of cancer cells. The RIG signaling pathway is also related to the development of cancer chemoresistance. For example, in recurrent or resistant ovarian cancer, RIG-I expression levels are significantly increased and are linked to poor prognosis [42]. Apart from that, RIG-I was reported to regulate the resistance of nasopharyngeal carcinoma to paclitaxel by regulating IFN/JAK2 [43]. In the current work, we found that TAFs derived exosomes can partially decrease the chemosensitivity to cisplatin both *in vitro and in vivo*, and this may achieve by the activation of the RIG-I/IFN-β signaling. These results suggested that TAFs derived exosomes may affect the chemosensitivity of TE-1 cells to cisplatin via RIG-I/IFN-β signaling.

## Conclusion

In this research, we investigated the function of TAFs-derived exosomes on ESCC cells. Our data showed that TAFs-exosomes promoted cell proliferation and cisplatin resistance via RIG-I/IFN-β axis. Our findings might represent a novel mechanism involved in cisplatin resistance of ESCC, and provide a new therapeutic strategy for ESCC chemoresistance.

## Author contributions

Yayun Cui: Writing-original draft, Investigation, Formal analysis, Data curation.

Shu Zhang: Perform supplementary experiments, Data curation.

Xiaohan Hu: Conceptualization, Formal analysis, Investigation.

Fei Gao: Conceptualization, Formal analysis, Writing-review and editing.

## Supplementary Material

Supplemental Material

## Data Availability

The data used to support the findings of this study are available from the corresponding author upon request.
